The article "Overexpression of SERCA2a Alleviates Cardiac Microvascular Ischemic Injury by Suppressing Mfn2-Mediated ER/Mitochondrial Calcium Tethering" was retracted in 2022. Reasons: compromised peer review; original data or images not available; concerns about the data.

# Overexpression of SERCA2a Alleviates Cardiac Microvascular Ischemic Injury by Suppressing Mfn2-Mediated ER/Mitochondrial Calcium Tethering

**DOI:** 10.3389/fcell.2021.636553

**Published:** 2021-04-01

**Authors:** Feng Tian, Ying Zhang

**Affiliations:** Department of Cardiology, The First Medical Center of PLA General Hospital, Beijing, China

**Keywords:** ischemia injury, hypoxia, mitochondria, CMEC, SERCA2a, Mfn2

## Abstract

Our previous research has shown that type-2a Sarco/endoplasmic reticulum Ca^2+^-ATPase (SERCA2a) undergoes posttranscriptional oxidative modifications in cardiac microvascular endothelial cells (CMECs) in the context of excessive cardiac oxidative injury. However, whether SERCA2a inactivity induces cytosolic Ca^2+^ imbalance in mitochondrial homeostasis is far from clear. Mitofusin2 (Mfn2) is well known as an important protein involved in endoplasmic reticulum (ER)/mitochondrial Ca^2+^ tethering and the regulation of mitochondrial quality. Therefore, the aim of our study was to elucidate the specific mechanism of SERCA2a-mediated Ca^2+^ overload in the mitochondria via Mfn2 tethering and the survival rate of the heart under conditions of cardiac microvascular ischemic injury. *In vitro*, CMECs extracted from mice were subjected to 6 h of hypoxic injury to mimic ischemic heart injury. C57-WT and Mfn2^KO^ mice were subjected to a 1 h ischemia procedure via ligation of the left anterior descending branch to establish an *in vivo* cardiac ischemic injury model. TTC staining, immunohistochemistry and echocardiography were used to assess the myocardial infarct size, microvascular damage, and heart function. *In vitro*, ischemic injury induced irreversible oxidative modification of SERCA2a, including sulfonylation at cysteine 674 and nitration at tyrosine 294/295, and inactivation of SERCA2a, which initiated calcium overload. In addition, ischemic injury-triggered [Ca^2+^]c overload and subsequent [Ca^2+^]m overload led to mPTP opening and ΔΨm dissipation compared with the control. Furthermore, ablation of Mfn2 alleviated SERCA2a-induced mitochondrial calcium overload and subsequent mito-apoptosis in the context of CMEC hypoxic injury. *In vivo*, compared with that in wild-type mice, the myocardial infarct size in Mfn2^KO^ mice was significantly decreased. In addition, the findings revealed that Mfn2^KO^ mice had better heart contractile function, decreased myocardial infarction indicators, and improved mitochondrial morphology. Taken together, the results of our study suggested that SERCA2a-dependent [Ca^2+^]c overload led to mitochondrial dysfunction and activation of Mfn2-mediated [Ca^2+^]m overload. Overexpression of SERCA2a or ablation of Mfn2 expression mitigated mitochondrial morphological and functional damage by modifying the SERCA2a/Ca^2+^-Mfn2 pathway. Overall, these pathways are promising therapeutic targets for acute cardiac microvascular ischemic injury.

The article "Overexpression of SERCA2a Alleviates Cardiac Microvascular Ischemic Injury by Suppressing Mfn2-Mediated ER/Mitochondrial Calcium Tethering" was retracted in 2022. Reasons: compromised peer review; original data or images not available; concerns about the data.

## Introduction

Acute myocardial infarction (AMI) refers to a clinical or pathological event with evidence of myocardial injury due to acute myocardial ischemia (Heusch, 2019; Kohlhauer et al., 2019). Although early coronary intervention and bypass surgery reduce the immediate mortality of patients, the incidence of long-term heart failure and recurrent myocardial infarction has still been increasing over time, creating a major disease burden to people worldwide (Hausenloy et al., 2020; Kleinbongard, 2020). Studies have shown that endothelial cells are affected earlier and are more sensitive to heart ischemia injury than cardiomyocytes (Singh et al., 2020; Wang et al., 2020a). Microcirculation injury is one of the most important pathological mechanisms of ischemic injury ([Bibr B62][Bibr B68]). Myocardial ischemic injury impairs the structure and function of endothelial cells, increases vascular tone, and leads to a decrease in cellular energy metabolism and ATP production (Bøtker, 2019; He et al., 2020). Thereby, it causes endothelial cell edema and mitochondrial damage, ultimately exacerbating myocardial damage. Therefore, preventing these adverse effects of heart ischemic injury on cardiac microvascular endothelial cell (CMEC) function is an important therapeutic strategy for cardio-protection.

Although researchers have revealed many mechanisms underlying ischemic injury (Gao et al., 2019; Bankapalli et al., 2020), the roles of calcium overload and subsequent oxidative stress in myocardial infarction injury are still far from clear (Basalay et al., 2020; Cao et al., 2020a). SERCA2a, the main factor involved in calcium handling, is an ATP-driven protein that transports Ca^2+^ back to the ER (Pinton et al., 2008). During cardiac infarction injury, the activity and expression of SERCA2a are reduced, leading to impaired cardiac contraction and diastolic function. Downregulation of SERCA2a expression is closely related to cytoplasmic calcium overload. Moreover, calcium overload leads to a large amount of ROS production and is closely related to the oxidative modification of SERCA2a (Temsah et al., 1999; Harrison et al., 2002; Singh et al., 2004). The adjacent tyrosine residues Tyr294 and Tyr295 are nitrated in skeletal muscle and cardiomyocytes of aged animals (Viner et al., 1999; Knyushko et al., 2005). Nitrification of tyrosine residues leads to decreased activity of SERCA2a (Lokuta et al., 2005; Mozaffarian et al., 2015). In myocardial samples from patients with dilated cardiomyopathy, nitrotyrosine modification of SERCA2a is positively correlated with abnormal cardiomyocyte function (Lokuta et al., 2005). These results indicate that the activity of SERCA2a is closely related to the oxidation state of cardiomyocytes. The antioxidant AON reduces the OPTM of SERCA2a, thereby improving SERCA2a activity (Mital et al., 2011). Given our interest in the role of oxidative stress in regulating Ca^2+^ handling and recent reports of OPTM of SERCA2a in models of heart disease (Viner et al., 1999; Knyushko et al., 2005; Lokuta et al., 2005; Mozaffarian et al., 2015), the effect of OPTM on SERCA2a after myocardial ischemic injury was evaluated in our present study.

The article "Overexpression of SERCA2a Alleviates Cardiac Microvascular Ischemic Injury by Suppressing Mfn2-Mediated ER/Mitochondrial Calcium Tethering" was retracted in 2022. Reasons: compromised peer review; original data or images not available; concerns about the data.

The mitochondrion, another important organelle involved in Ca^2+^ storage in cells, regulates intracellular and mitochondrial Ca^2+^ homeostasis. Mitochondria uptake calcium during acute ischemic injury via a calcium uniporter from the SR and induce MPTP opening at the beginning of oxygen shortage, which is the main determinant of myocardial cell death (Ruiz-Meana et al., 2009). Recent studies have shown that Mfn2 acts as a fusion protein in the mitochondrial outer membrane and plays an important role in Ca^2+^ transfer from the SR to mitochondria. Moderate mitochondrial/SR tethering is essential for maintaining cardiac bioenergetics. However, a large amount of Ca^2+^ transport to the mitochondria activates mitophagy and ROS signaling (Eksborg, 1989; Hu et al., 2016). There are two subtypes of mitochondrial fusion proteins: Mfn1 and Mfn2. Ablation of both Mfn1 and Mfn2 conferred resistance to ischemic stress-induced mPTP opening or impaired mitochondria/SR tethering and contributed to the protective effects (de Brito and Scorrano, 2008; Papanicolaou et al., 2011, 2012a). However, the long-term effects of ablating these proteins are detrimental and have been shown to cause cardiomyopathy and sudden cardiac death (Chen et al., 2011). How Mfn2 mediates cardioprotective or detrimental effects, especially in CMECs, is still unknown. Ca^2+^ acts as an important signaling molecule in heart infarct injury. It is transferred from the cytoplasm to the SR by SERCA2a and further transferred from the SR to mitochondria via Mfn2 tethering. Deficiency of Mfn2 substantially reduced Ca^2+^ transfer from the SR to the mitochondria (Bonora et al., 2015). However, the specific mechanisms underlying the interaction between SERCA2a and Mfn2 need to be clarified.

Therefore, the aim of our study was to further characterize the role of Mfn2 in CMECs in a model of ischemic injury. In this study, by using Mfn2^KO^ mice, we clearly demonstrated that SERCA2a-dependent [Ca^2+^]c overload leads to mitochondrial dysfunction and activation of Mfn2-mediated [Ca^2+^]m overload. Mfn2, a downstream target of SERCA2a, activates Drp-1-dependent mito-fission and subsequently Parkin/PINK-dependent mitophagy.

The article "Overexpression of SERCA2a Alleviates Cardiac Microvascular Ischemic Injury by Suppressing Mfn2-Mediated ER/Mitochondrial Calcium Tethering" was retracted in 2022. Reasons: compromised peer review; original data or images not available; concerns about the data.

## Materials and Methods

### Animal Model of Cardiac Ischemic Injury *in vivo*

All animal procedures were approved by the Chinese PLA General Hospital Animal Care and Use Committee and were in accordance with the Guide for the Care and Use of Laboratory Animals (published by the US National Institutes of Health, NIH Publication No. 85-23, revised 1996). The Mfn2 loxp/loxp mice with cardiomyocyte-specific deletion of the mfn2 exon were generated based on the Cre-Lox strategy (Baines et al., 2005; Zheng et al., 2009; Dai et al., 2011). Briefly, exon 4 of Mfn2 was knocked out by homologous recombination, and the gene exons were combined with myh6-driven nuclear-localized Cre to generate cardiac-specific Mfn2 knockout mice (Mfn2^KO^). All mice were bred on a C57BL/6 background for at least 3 generations. Subsequently, 8-week-old wild-type (WT) and Mfn2^KO^ mice were used to establish a heart ischemic injury model according to our previous studies with minor modifications (Zhou et al., 2020). For the heart ischemia procedure, the mice were anesthetized with isoflurane, and the hearts were exposed via a left thoracotomy. The left anterior descending coronary artery (LAD) was ligated by 7–0 silk sutures for 1 h to mimic ischemic conditions. After that, blood was collected to measure myocardial enzyme markers such as LDH, troponin T, and CK-MB using ELISA. Infarct size was measured using Evans blue and TTC methods in different groups (Lustgarten Guahmich et al., 2020).

### Cardiac Microvascular Endothelial Cell Extraction From Mice and Adenovirus Vector Transfection

CMECs were isolated from C57BL/6 background WT mice (6 months old) using the enzyme dissociation method as previously reported with minor modifications (Zhou et al., 2018). In brief, mice were euthanized using isoflurane under sterile conditions. After removing the atria, the right ventricles, and the outer membrane or other tissues, left ventricle tissues were immersed in 75% ethanol for 15 s. The remaining tissue was digested in 0.2% (w/v) collagenase type I for 10 min and subsequently in 0.25% (w/v) trypsin for 5 min at 37°C. The samples were further resuspended in Dulbecco’s modified Eagle’s medium (DMEM) containing 20% (v/v) fetal bovine serum (FBS) (Pflüger-Müller et al., 2020).

The SERCA2a gene adenoviral vector was used to overexpress SERCA2a in CMECs. A non-cell-type-specific recombinant adenovirus vector carrying the SERCA2a gene (Ad-SERCA2a, stock in 1 × 1010 PFU/ml) and an empty recombinant adenovirus vector (Ad-ctrl, stock in 1.9 × 1010 PFU/ml) were constructed using the vector gene technique. Synthetic SERCA2a gene adenovirus vectors were injected by Hua Yueyang Biotechnology Co., Ltd. (Beijing, China). Next, we established siRNA-Mfn2 in CMECs (Pabel et al., 2020). Twenty-four hours before transfection, the cells were seeded in six-well plates until the cell confluence reached approximately 50%, at which time the CMECs were transfected with Lipofectamine 2000 (Invitrogen, CA, United States). Subsequently, the above reagent was mixed and incubated at room temperature for 20 min. The mixture was cultured in a 5% CO_2_ incubator at 37°C for 6–8 h. The subsequent experiment was conducted after the cells had been cultured for 24–48 h. A synthetic Mfn2 gene fragment was introduced by Hua Yueyang Biotechnology Co., Ltd. (Biotechnology Co., Beijing, China). Two sets of Mfn2-siRNA were designed and had the following sequences: 5′-GGACCCAGTTACTACAGAAGA-3′ and 5′-GCTCCTGGCTCAAGACTATAA-3′. The control gene was UUCUCCGAACGUGUCACGUTT (primer sequences: 5′–3′).

The article "Overexpression of SERCA2a Alleviates Cardiac Microvascular Ischemic Injury by Suppressing Mfn2-Mediated ER/Mitochondrial Calcium Tethering" was retracted in 2022. Reasons: compromised peer review; original data or images not available; concerns about the data.

### *In vitro* Hypoxic Injury Model in Cardiac Microvascular Endothelial Cells

CMECs were extracted from C57BL/6 WT mice to establish a hypoxic injury model *in vitro* as previously described (Zhang et al., 2016). Briefly, 95% concentrated N_2_ and 5% CO_2_ were mixed in a tri-gas incubator, and the CMECs were cultured for approximately 6 h. Next, the cells were changed to normal DMEM (high glucose, Gibco, United States) containing 5% fetal bovine serum (FBS, HyClone, United States) at 37°C to perform further experiments immediately (Lindner et al., 2020).

### Detection of Cytoplasmic and Mitochondrial Ca^2+^ and ROS Levels and Cell TUNEL Assay

Cells were incubated with Fluo-3 AM (S1056, Beyotime) or Rhod-2 (Abcam, ab142780) for 30 min. After washing with PBS, the intensities of cytoplasmic Ca^2+^ and mito-Ca^2+^ were detected by flow cytometry (Sysmex Partec GmbH, Germany) and immunofluorescence using a Leica confocal microscope (Leica, Wetzlar, Germany). Cytoplasmic ROS was measured by DCFH-DA (Sigma) (Domingues et al., 2020). ImageJ was used to assess fluorescence intensity (Fluo-3, Rhod2, and TMRM). Data (F/F0) were obtained by dividing the fluorescence intensity (F) by (F0) at the resting level (*t* = 0), which was normalized by the control group. The TUNEL assay was used according to the manufacturer’s instructions to detect cell death after hypoxic injury. For quantification, the numbers of TUNEL-positive cells were calculated in at least 10 random separate fields to obtain the average percentage in different groups (di Somma et al., 2020).

The article "Overexpression of SERCA2a Alleviates Cardiac Microvascular Ischemic Injury by Suppressing Mfn2-Mediated ER/Mitochondrial Calcium Tethering" was retracted in 2022. Reasons: compromised peer review; original data or images not available; concerns about the data.

### Isolation of Sarcoplasmic Reticulum Microsomes and Measurement of Sarco/Endoplasmic Reticulum Ca^2+^-ATPase Activity and MDA, GPX, and SOD Levels

Briefly, isolated hearts were homogenized in buffer containing 10 mM imidazole (pH 7.0), 300 mM sucrose, 1 mM EDTA, 1 mM or 10 mM DTT and 0.3 mM phenylmethylsulfonyl fluoride. Homogenates were centrifuged at 8,000 g for 20 min. The supernatant was removed, adjusted to a final concentration of 600 mM and centrifuged at 100,000 g for 1 h. The pellet was resuspended in homogenization buffer with 600 mM NaCl and centrifuged again at 100,000 g for 1 h (Adapala et al., 2020). The pellet was resuspended in homogenization buffer without DTT. Then, the samples were incubated with a final concentration of 100 μM urea peroxide for 20 min on ice, and the urea peroxide was subsequently neutralized by DTT. SR microsomal protein content was quantified via the Bradford method. The supernatants from cells or tissues were collected to perform ELISA to measure SERCA2a activity and MDA, GPX, SOD, MCP-1, TNFα, and IL-6 levels in different groups according to the manufacturer’s instructions (Lamas Bervejillo et al., 2020).

### Isolation of Cardiac Mitochondria, mPTP Opening Assay, and JC-1 Staining

CMEC mitochondria were isolated as described previously (Amiott et al., 2008). The mPTP opening assay was performed via an established calcein cobalt loading procedure by incubating cells with calcein-acetoxymethylester (calcein-AM) according to a previous study (Shi et al., 2018). The immunofluorescence intensity of calcein-AM was measured to assess mPTP opening. The mitochondrial potential was observed by incubating the cells with the JC-1 probe (1.10 mg/ml) for 30 min at 37°C in the dark. After washing three times with PBS, the cells were then observed under a fluorescence microscope (Kremslehner et al., 2020).

### Co-immunoprecipitation

After treatment, the samples were precleaned with Protein A/G (Santa Cruz Biotechnology) and incubated with antibodies as follows. Then, Protein A/G was added, and the samples were shaken at 4°C overnight. The precipitates were washed three times with PBS, and the proteins were denatured for Western blot analysis. The primary antibodies were anti-nitrotyrosine (NT) (1:200; Santa Cruz Biotechnology) and anti-SERCA2a (1:1,000; Abcam, #ab3625) (Cuijpers et al., 2020). The methods used to develop the antibody directed at SERCA2a sulfonylated at cysteine 674 were previously described (Xu et al., 2006). The peptides were chemically synthesized with constituent amino acids, including nitrotyrosine. Each antigen was injected into rabbits, and serum was obtained approximately every 2 weeks. To remove antibodies to the non-sulfonylated sequences, antisera were processed over immunosorbents consisting of non-sulfonylated peptides immobilized on agarose. Subsequently, the specific antibody against the sulfonylated cysteine peptide was column purified from the processed antisera by using immunosorbents consisting of the sulfonylated peptide immobilized on agarose. Yields of antibody ranged from 10 to 30 μg/ml. The sulfonylated cysteine concentration used in the experiment was 20 μg/ml (Cao et al., 2020b).

The article "Overexpression of SERCA2a Alleviates Cardiac Microvascular Ischemic Injury by Suppressing Mfn2-Mediated ER/Mitochondrial Calcium Tethering" was retracted in 2022. Reasons: compromised peer review; original data or images not available; concerns about the data.

### Colocalization of Immunofluorescence Staining

SERCA2a and Mfn2 expression was assessed by immunofluorescence staining. Briefly, cells were collected and fixed with 4% paraformaldehyde for 10 min, permeabilized with 0.5% Triton X-100 for 10 min, and blocked with 10% goat serum albumin (Invitrogen, United States) for 1 h at room temperature (Vitturi et al., 2020). Subsequently, the samples were incubated with primary antibodies overnight at 4°C, washed with PBS three times, and incubated with secondary antibody for 45 min at room temperature. Finally, DAPI (Sigma-Aldrich, United States) was added, and the cells were analyzed under a fluorescence microscope.

### Electron Microscopy and Echocardiography Measurements

Echocardiography was immediately performed in all mice after the heart ischemia model was established. Left ventricular fraction shortening (LVFS), left ventricular ejection fraction (LVEF), left ventricular dilated dimension (LVDD) and left ventricular volume-systole (LVV) were measured in M-mode images using computer algorithms (Tan et al., 2020a).

The microvascular ultrastructure in the heart was evaluated using electron photomicrographs (EM). Heart samples were fixed in 5% glutaraldehyde and 4% paraformaldehyde in 0.1 M sodium cacodylate buffer (pH 7.4) with 0.05% CaCl_2_ for 24 h. After washing in 0.1 M sodium cacodylate buffer, tissues were postfixed in 1% OsO4 and 0.1 M cacodylate buffer overnight, dehydrated and embedded in Embed 812 resin (Zhang et al., 2020). The sections were stained with 2% uranyl acetate followed by 0.4% lead citrate and viewed with a Philips 400 electron microscope (Electron Microscopy Sciences).

### Western Blot and Reagent Treatment

Briefly, tissues were homogenized and sonicated in lysis buffer. Next, the samples were centrifuged for approximately 10 min at 4°C to obtain the supernatants. Equivalent amounts of protein from different groups were separated by SDS-PAGE and subsequently transferred to a polyvinylidene difluoride (PVDF) membrane (Latacz et al., 2020). The membranes were incubated with the following primary antibodies at 4°C overnight: anti-SERCA2a (1:1,000; Abcam, #ab3625), GAPDH (1:1,000, Abcam, #ab8245), Actin (1:1,000, sc-1616, Santa Cruz Biotechnology), Parkin (1:1,000, Abcam, #ab77924), p62 (1:1,000, Abcam, #ab101266), pink1 (1:1,000, Abcam, #ab23707), Bcl-2 (1:1,000, Abcam, #ab32124), Bax (1:1,000, Abcam, #ab18283), VDAC (1:1,000, Abcam, #ab15895), Mfn2 (1:1,000, Abcam, #ab56889), Cyt-C (1:1,000, Abcam, #ab13575), Caspase9 (1:1,000, Abcam, #ab32539), Cle-Caspase3 (1:1,000, Cell Signaling Technology, #9664), Drp-1 (1:1,000, Abcam, #ab56788), and Fis-1 (1:1,000, Abcam, #ab229969). Then, the membranes were incubated with secondary antibodies at room temperature for 1 h. Band intensity was quantified using Image-Pro Plus 6.0 software.

The article "Overexpression of SERCA2a Alleviates Cardiac Microvascular Ischemic Injury by Suppressing Mfn2-Mediated ER/Mitochondrial Calcium Tethering" was retracted in 2022. Reasons: compromised peer review; original data or images not available; concerns about the data.

All cell groups were treated in serum-containing Dulbecco’s modified Eagle’s medium and starved for at least 16 h. To determine the effect of cytosolic Ca^2+^, the cell-permeable Ca^2+^ chelator BAPTA (Sigma) was used before the injury model. To detect the effect of ROS levels on different groups of CMECs, NAC (Sigma) was used as the negative group. tBHQ (Sigma) was used as a pretreatment to inhibit the expression of SERCA2a (Ko et al., 2020). To confirm the function of mito-fission, CCCP (Sigma) was used to induce spontaneous damaged fission.

### Immunohistochemistry and Hematoxylin and Eosin Staining

Tissues were immersed in 4% paraformaldehyde for 4 h and transferred to 70% ethanol. Then, the tissues were placed in cassettes, dehydrated through a serial alcohol gradient, and embedded in paraffin wax blocks. Histopathological examination was performed in infarcted tissue on formalin-fixed, paraffin-embedded 5–6 μm sections stained with hematoxylin and eosin using standard methods and examined via light microscopy (Mak et al., 2020). Primary antibodies against CD68 (1:500, Abcam, #ab31630) and eNOS (1:300, Abcam, #ab76198) were used. A TUNEL assay kit was used according to the manufacturer’s instructions (R&D Systems). HE staining was used to detect the arrangement of RBC morphology to evaluate the integrity of microvessels.

### Statistical Analysis

Data are expressed as the mean ± SEM. Statistical comparisons were performed using two-tailed non-paired *t*-tests to evaluate different groups. For comparisons among more groups, one-way ANOVA was used, and statistical significance was set at *p* < 0.05.

## Results

Hypoxic injury induced oxidative posttranslational modification of SERCA2a and triggered cytoplasmic Ca^2+^ imbalance. We extracted CMECs from C57/WT mice and established a 6 h hypoxia injury model *in vitro*. SERCA2a is the main ATP-dependent protein that returns Ca^2+^ to the endoplasmic reticulum to balance cytoplasmic free Ca^2+^. A calcium map was used to quantitatively analyze the change in [Ca^2+^]c (cytoplasmic calcium) in different groups. As shown in Figures 1A,B, the data demonstrated that hypoxic injury significantly increased [Ca^2+^]c intensity, while this effect was blocked by SERCA2a overexpression or pretreatment with the antioxidant reagent NAC. To confirm the effect of elevated Ca^2+^ levels on cell survival, we performed a TUNEL assay, and the results showed that there were more cell deaths in the hypoxic injury group than in the control group (Figures 1C–E). Compared with hypoxic injury, overexpression of SERCA2a or treatment with NAC reagent reduced the ratio of TUNEL-positive cells, indicating that mitigation of [Ca^2+^]c overload had an antiapoptotic effect on CMEC hypoxic injury. A previous report indicated that cellular oxidative stress might inactivate SERCA2a and subsequently induce [Ca^2+^]c imbalance. Furthermore, DCFH-DA showed that hypoxic injury increased the fluorescence intensity, while overexpression of SERCA2a or NAC reagent reduced the oxidative stress level to some extent. These results were consistent with the ELISA results for MDA, GPX, and SOD levels (Figures 1F–I). Previous research found oxidative cysteine modification of SERCA2a under oxidative conditions. In our present study, we used Western blot and immunoprecipitation assays to evaluate irreversible oxidative modifications of SERCA2a consisting of sulfonylation at cysteine 674 and nitration at tyrosines 294/295. We developed antibodies directed at SERCA2a sulfonylated at cysteine 674 and SERCA2a nitrated at tyrosine 294/295. The specific methods are described in the materials. Immunoprecipitation assays revealed that (Figures 1J–M) the hypoxia group showed higher staining of SERCA2a sulfonylated at cysteine 674 and SERCA2a nitrated at tyrosine 294/295 than the control group. However, overexpression of SERCA2a or treatment with the antioxidant reagent NAC significantly and irreversibly decreased sulfonylated and nitrated SERCA2a expression.

The article "Overexpression of SERCA2a Alleviates Cardiac Microvascular Ischemic Injury by Suppressing Mfn2-Mediated ER/Mitochondrial Calcium Tethering" was retracted in 2022. Reasons: compromised peer review; original data or images not available; concerns about the data.

**FIGURE 1:** Hypoxic injury-induced oxidative modification of sarco/endoplasmic reticulum CSERCA2a and SERCA2a-induced Ca^2+^ imbalance (*n* = 3/group). **(A,B)** A calcium map was used to quantitatively analyze the change in [Ca^2+^]c (cytoplasmic calcium) in the different groups. **(C–E)** TUNEL assays and DCFH-DA fluorescence were used to assess cell survival. **(F–I)** ELISA results showing the changes in MDA, GPX, and SOD levels and the activity of SERCA2a after hypoxic injury in CMECs. **(J–M)** The relative expression levels of SERCA2a with nitrotyrosine and SERCA2a with sulfonylated cysteine were assessed by coimmunoprecipitation assays. *p < 0.05 compared with the Ad-Ctrl; ^#^*p* < 0.05 compared with the Hypo(Ad-Ctrl).

Excessive [Ca^2+^]c triggered by oxidative modification of SERCA2a was demonstrated to be a critical factor involved in cell apoptosis, while overexpression of SERCA2a attenuated reperfusion-induced oxidative stress. Another free Ca^2+^ storage organelle, the mitochondrion ([Ca^2+^]m), can be filled with excessive Ca^2+^, resulting in [Ca^2+^]m overload and serious side effects. Therefore, we hypothesized that in CMECs with hypoxic injury, [Ca^2+^]m overload would be followed by pathologically excessive [Ca^2+^]c levels. First, we used the [Ca^2+^]m probe Fluo-3AM and the [Ca^2+^]c probe Rhod2 to detect the change in Ca^2+^ concentration in different groups by flow cytometry (Figures 2A–D). Under hypoxic conditions, either [Ca^2+^]c or [Ca^2+^]m significantly increased compared to that under control conditions, while overexpression of SERCA2a caused both [Ca^2+^]c and [Ca^2+^]m to decrease to some extent. Pretreatment with the cytoplasmic Ca^2+^ chelator BAPTA largely neutralized [Ca^2+^]c, while the use of BAPTA had no obvious effect on [Ca^2+^]m, suggesting that [Ca^2+^]c was transported to the mitochondria in this specific way. To further observe the effect of [Ca^2+^]m overload on the function of the mitochondria (Figures 2E–H), we used JC-1 staining to detect damage to the mitochondrial membrane potential (ΔΨm) and the opening of the mitochondrial permeability transition pore (mPTP), which are prerequisites for mitochondrial inner membrane protein release. The results indicated that hypoxic injury-induced [Ca^2+^]c and [Ca^2+^]m overload finally led to increased mPTP opening and dissipated ΔΨm compared with those in the control group. However, overexpression of SERCA2a or pretreatment with BAPTA recovered the function of mitochondria to some extent.

**FIGURE 2:** Excessive [Ca^2+^]m was followed by SERCA2a-dependent [Ca^2+^]c overload and mitochondrial dysfunction (*n* = 3/group). **(A–D)** The [Ca^2+^]m probe Fluo-3AM and the [Ca^2+^]c probe Rhod2 were detected by flow cytometry to assess changes in Ca^2+^ concentration in the different groups. **(E–H)** The change in membrane potential (ΔΨm) was detected by JC-1 staining. The arbitrary mitochondrial permeability transition pore (mPTP) opening time was determined as the time when the TMRE fluorescence intensity decreased by half between the initial and final fluorescence intensities. *p < 0.05 compared with the Ad-Ctrl; ^#^*p* < 0.05 compared with the Hypo(Ad-Ctrl).

Based on the results above, we hypothesized that [Ca^2+^]c was transported to mitochondria via Ca^2+^ channels. Research has indicated that despite apparent mitochondrial dysfunction, hearts deficient in Mfn2 are protected against acute myocardial infarction due to impaired mitochondria/SR tethering (Hall et al., 2016). However, the role of Mitofusin2 in the context of microvessel damage in acute myocardial infarction injury is unclear. Therefore, we wondered whether SERCA2a-dependent Ca^2+^ imbalance is an upstream target of Ca^2+^ mitochondria/SR tethering. First, Western blotting was used to observe Mfn2 expression in different groups (Figures 3A,B). The results showed that Mfn2 expression was obviously increased in the hypoxia group compared to the control group, while overexpression of SERCA2a or pretreatment with BAPTA downregulated the level of Mfn2. Based on the results of SERCA2a overexpression, we used the SERCA2a inhibitor tBHQ to block the benefit of SERCA2a-Ca^2+^ recycling. The results showed that after inhibition of SERCA2a, the expression of Mfn2 increased, which verified that Mfn2 is a downstream target of SERCA2a. The results were further proven by coimmunofluorescence staining of SERCA2a and Mfn2 (Figures 3C,D). The intensity of SERCA2a fluorescence was decreased in the context of hypoxic injury, and Mfn2 fluorescence was elevated. However, overexpression of SERCA2a or treatment with BAPTA reversed this change. To further detect the impact of Mfn2 on mitochondrial function, we established gene silencing technology to knock down the expression of Mfn2 (siMfn2), and the knockdown efficiency was proven by WB assay. Then, we used the [Ca^2+^]c probe Fluo-3 and the [Ca^2+^]m probe Rhod2 to observe the changes in Ca^2+^ concentrations (Figures 3E,F). In CMECs with hypoxic injury, a higher [Ca^2+^]c concentration paralleled the content of [Ca^2+^]m. However, overexpression of SERCA2a or removal of free Ca^2+^ by BAPTA treatment led to a significant decrease in [Ca^2+^]m in CMECs with hypoxic injury. Furthermore, inhibition of Mfn2 had no effect on [Ca^2+^]c, but it inhibited [Ca^2+^]m overload, which indicated that Mfn2 was a critical channel for [Ca^2+^]c inflow into mitochondria. These results suggested that the elevated function of Mfn2 under oxygen deficiency conditions was the main cause of [Ca^2+^]m overload, while SERCA2a was able to suppress Mfn2 expression by regulating Ca^2+^ balance. It is well known that in addition to organelle tethering, Mfn2 is also located in the mitochondrial outer membrane and participates in Parkin-mediated mitophagy to remove damaged mitochondrial fragments. To further determine the impact of SERCA2a overexpression and Mfn2 knockdown on mitochondrial function and mitophagy, we first used electron microscopy to observe autophagosome formation (Figure 3I). The results indicated that autophagosome activity was much higher under hypoxic heart injury conditions than under control conditions. However, overexpression of SERCA2a or knockdown of Mfn2 obviously decreased autophagosome activity. To determine the underlying mechanism, we extracted proteins from the mitochondrial fraction and cytoplasm to compare the changes in mitophagy-related proteins. We found that Parkin/PINK-dependent mitophagy was significantly activated in the hypoxia model, while blocking the expression of Mfn2 not only decreased Ca^2+^ flow into mitochondria but also weakened the ability of Parkin/PINK-dependent mitophagy to remove damaged mitochondrial fragments in the context of hypoxic injury. Then, Western blotting was performed to determine the effect of Mfn2 knockdown on the balance of mitochondrial quality (Figures 3G,H). The data suggested that the Cyt-C protein entered the cytoplasm, and mito-apoptosis-related proteins, such as Bax, caspase 9, and caspase 3, were activated in the hypoxic pretreatment group. However, overexpression of SERCA2a or knockdown of Mfn2 reversed mitochondria-induced apoptosis to some extent. These results illustrated that even though the knockdown of Mfn2 inhibited the ability of mitophagy to clear damaged mitochondrial fragments, overexpression of SERCA2a or knockdown of Mfn2 also benefited the balance of mitochondrial quality and the survival of CMECs.

The article "Overexpression of SERCA2a Alleviates Cardiac Microvascular Ischemic Injury by Suppressing Mfn2-Mediated ER/Mitochondrial Calcium Tethering" was retracted in 2022. Reasons: compromised peer review; original data or images not available; concerns about the data.

**FIGURE 3:** SERCA2a-dependent [Ca^2+^]c overload activated mitofusin 2 (Mfn2)-mediated [Ca^2+^]m overload and was accompanied by increased Parkin/PINK-dependent mitophagy (*n* = 3/group). **(A,B)** Western blot analysis was performed to detect the expression of Mfn2. Hypoxia and pretreatment with tBHQ increased the expression of Mfn2, while overexpression of SERCA2a, pretreatment with BAPTA and knockdown of the Mfn2 gene reversed the Mfn2 expression level. **(C,D)** Coimmunofluorescence of SERCA2a and Mfn2 in cardiac microvascular endothelial cells (CMECs). The overlap of fluorescence intensity changed in the different groups and was consistent with the changes observed in WB. **(E,F)** The [Ca^2+^]c probe (Fluo-3) and [Ca^2+^]m probe (Rhod2) were used to observe changes in Ca^2+^ concentration via fluorescence. **(G,H)** Western blot analysis was performed to detect Parkin/PINK-dependent mitophagy- and mito-apoptosis-related protein expression in the different groups. **(I)** Electron microscopy was used to observe autophagosome formation. *p < 0.05 compared with the Ad-Ctrl; ^#^*p* < 0.05 compared with the Hypo(Ad-Ctrl).

### SERCA2a-Dependent [Ca^2+^]c Overload Triggered Mfn2-Mediated [Ca^2+^]m Overload and Was Accompanied by Increased Drp-1-Dependent Mitochondrial Fission

Previous studies have indicated that [Ca^2+^]m overload not only triggers calcium imbalance but is also accompanied by mito-oxidative stress. Therefore, a reactive oxygen probe was used to detect mitochondrial ROS activity. The results indicated that the ROS activity of the hypoxic injury group was 4-fold higher than that of the control group, while overexpression of SERCA2a or knockdown of Mfn2 significantly decreased the ROS activity in mitochondria (Figures 4A,B). Moreover, after constructing the damage model, mitochondria were extracted from the cells and used for ATP content and glucose uptake tests (Figures 4C,D). Furthermore, the supernatant was collected after hypoxic injury modeling in CMECs, and lactate production was analyzed using ELISA (Figure 4E). The results showed that cardiac injury caused obviously decreased ATP production and glucose uptake, while overexpression of SERCA2a or knockdown of Mfn2 improved mitochondrial energy generation and metabolic function. Our previous studies have proven that excessive mito-oxidative stress induces fatal mitochondrial fission. In this study, we wondered whether the function of SERCA2a or the downstream factor Mfn2 also affects mitochondrial fission activity. First, we designed our experiment by performing coimmunofluorescence staining of mitochondrial morphology and lysosomes (Figures 4F,G). In the hypoxic injury group, the length of mitochondria was obviously decreased compared with that in the control group; the hypoxic injury group also showed elevated diffuse lysosome fluorescence that overlapped with the fragmented mitochondria. This conclusion was also supported by pretreatment with the mito-fission activator CCCP, which showed the same effect as hypoxic injury. Overexpression of SERCA2a, knockdown of Mfn2, and treatment with the Ca^2+^ chelator BAPTA seemed to be effective ways to restore the normal morphology of mitochondria. During follow-up experiments (Figures 4H,I), we further proved by Western blot analysis that mito-fission activity was dependent on Drp-1 and Fis-1 protein expression. Therefore, we elucidated that the mechanism of cardiac hypoxic injury was Mfn2-mediated [Ca^2+^]m overload-triggered mitochondrial oxidative damage, which increased Drp-1-dependent mitochondrial fission and was accompanied by subsequent mitophagy activity to remove mitochondrial fragments.

The article "Overexpression of SERCA2a Alleviates Cardiac Microvascular Ischemic Injury by Suppressing Mfn2-Mediated ER/Mitochondrial Calcium Tethering" was retracted in 2022. Reasons: compromised peer review; original data or images not available; concerns about the data.

**FIGURE 4:** SERCA2a-dependent [Ca^2+^]c overload triggered Mfn2-mediated [Ca^2+^]m overload and was accompanied by increased Drp-1-dependent mitochondrial fission (*n* = 3/group). **(A,B)** A Mito-ROS probe (MitoSOX) was used to compare the mito-oxidative stress levels between the different groups. **(C–E)** ELISA and tests on extracted mitochondria were performed to detect the function of mitochondria in the different groups. **(F,G)** Coimmunofluorescence of mitochondria and lysosomes in CMECs. The overlap of fluorescence intensity changed in the different groups to reveal the morphology of mitochondria and the function of lysosomes. **(H,I)** Western blot analysis was performed to detect Drp-1- and Fis-1-dependent mito-fission expression in different groups. *p < 0.05 compared with the Ad-Ctrl; ^#^*p* < 0.05 compared with the Hypo(Ad-Ctrl); ^&^*p* < 0.05 compared with the Hypo(Ad-SERCA).

Based on the results of our *in vitro* experiments, in CMECs we next conducted a 1-h LAD ligation experiment to mimic myocardial ischemia *in vivo* in C57-WT mice and Mfn2^KO^ mice. Infarction areas were quantified in the different groups (Figures 5A,B) and showed that the cardiac ischemic injury model was established successfully and that Mfn2^KO^ significantly decreased the infarct size (ischemic group 42.3 ± 4.5% vs. Mfn2^KO^ group 21.9 ± 2.4%, *p* < 0.05). Furthermore, we used qPCR to test the efficiency of Mfn2 knockout in mice (Figure 5C). Then, immunohistochemical assays showed that the percentage of TUNEL-positive cells around the infarcted tissue in the ischemic group was much higher than that in the control group, and Mfn2^KO^ decreased the percentage of TUNEL-positive cells (ischemic group 53.8 ± 5.6% vs. Mfn2^KO^ group 28.6 ± 5.5%, *p* < 0.05) (Figures 5D,E). Moreover, the results were consistent with those of the WB analysis of the apoptosis-related proteins caspase9 and Cle-caspase3 in the corresponding groups (Figures 5F,J). As shown in Figures 5G–I, acute heart infarction indicators, such as LDH, Troponin T, and CK-MB, were significantly elevated after ischemic injury and downregulated in the Mfn2^KO^ mice. Echocardiography was performed to further assess heart contraction function, and the results showed that the ischemic injury mice had obvious evidence of impaired myocardial contractile function, including reduced ejection fraction, fractional shortening, increased LVDD and enlarged LV-systolic volume (Figures 5K–N), while these indicators were improved in Mfn2^KO^ mice under ischemic injury conditions. These data illustrated that cardiac ischemic injury led to severely damaged cardiac tissue and impaired heart contractile function, which might be related to dysfunction of the Mfn2 protein.

**FIGURE 5:** Knockdown of Mfn2 decreased heart infarction under cardiac ischemic injury conditions (*n* = 3/group). **(A,B)** Representative images of heart sections with TTC and Evans Blue staining of the infarcted area. The bar graph indicates the infarct size (ischemia group 42.3 ± 4.5% vs. Mfn2^KO^ group 21.9 ± 2.4%, *p* < 0.05). **(C)**. qPCR was used to test the efficiency of Mfn2 knockout in the Mfn2^KO^ mice. **(D,E)** The ischemic injury group presented more TUNEL-positive cells than the sham group. **(F,**J) Western blot analysis was performed to detect apoptosis-related protein expression in different groups. **(G–I)** ELISA analysis found significantly higher levels of LDH, troponin T, and CK-MB after ischemic injury, while the Mfn2^KO^ group showed some reversal of these effects. **(K–N)** Representative M-mode echocardiograms were performed after 1 h of heart ischemic injury in each group, and quantitative analysis of the cardiac data derived from echocardiograms was performed. *p < 0.05 compared with the Sham(WT); ^#^*p* < 0.05 compared with the Ische(WT).

The article "Overexpression of SERCA2a Alleviates Cardiac Microvascular Ischemic Injury by Suppressing Mfn2-Mediated ER/Mitochondrial Calcium Tethering" was retracted in 2022. Reasons: compromised peer review; original data or images not available; concerns about the data.

### Mfn2 Knockdown Attenuated Cardiac Microcirculatory Ischemic Injury

Electron microscopy of the heart infarction area revealed predominantly fragmented interfibrillar mitochondria (severe swelling or rupture) (Figure 6A). However, even though the morphological structure of mitochondria in Mfn2^KO^ mice was improved compared with that in WT ischemic injury mice, the Mfn2^KO^ mice still showed obvious fragmentation and swelling of mitochondria similar to that in the WT mice. Ischemic injury mice displayed abnormal red blood cell (RBC) morphology (the control RBCs were parachute-shaped), which indicated severe damage to microvessel integrity and barrier function (Figure 6B). To assess the integrity of microvessels, we conducted immunohistochemical staining (Figures 6C–E). In the ischemic injury mice, the data showed decreased release of eNOS from microcirculatory endothelial cells and large dispersed CD8-positive inflammatory cells, whereas the damaged microvessels in the Mfn2^KO^ mice recovered to some extent. Furthermore, blood was collected after cardiac ischemic injury, and the concentrations of inflammatory factors (MCP-1, TNFα, and IL-6) were analyzed using ELISAs, which indicated that ischemic injury induced higher inflammatory reactions (Figures 6F–H). However, the increased inflammatory factors in tissues were reversed by Mfn2^KO^.

**FIGURE 6:** Knockdown of Mfn2 attenuated cardiac microcirculatory ischemic injury (*n* = 3/group). **(A)** Electron microscopy revealed fragmented interfibrillar mitochondria. **(B)** HE staining for red blood cell morphology and arrangement among heart microcirculation in the different groups. **(C–E)** Immunohistochemistry of CD68 and eNOS expression in endothelial cells was performed to assess the integrity of microvessels in the different groups. **(F–H)** Blood was collected after cardiac ischemic injury, and the concentrations of inflammatory factors in the different groups were analyzed using MCP-1, TNF, and IL-6 ELISAs. *p < 0.05 compared with the Sham(WT); ^#^*p* < 0.05 compared with the Ische(WT).

The article "Overexpression of SERCA2a Alleviates Cardiac Microvascular Ischemic Injury by Suppressing Mfn2-Mediated ER/Mitochondrial Calcium Tethering" was retracted in 2022. Reasons: compromised peer review; original data or images not available; concerns about the data.

## Discussion

Cardiac AMI still has high mortality and rehospitalization rates because of delayed diagnosis and treatment, the high risk associated with intervention and surgery, and poor prognosis, especially in aging AMI patients (Cassar et al., 2009). Therefore, it is still urgent to explore the mechanisms underlying ischemic injury to provide effective prevention and treatment for AMI patients (Miyazaki et al., 2011; Pan et al., 2011). The ER is responsible for the synthesis, modification, folding, and transport of secreted proteins and for regulating intracellular Ca^2+^ homeostasis. It is highly sensitive to the loss of cellular energy and redox status and changes in cytosolic Ca^2+^ concentration, which ultimately lead to the accumulation of unfolded proteins, a condition known as ER stress (Okada et al., 2004; Yang et al., 2012). Ca^2+^ is a key molecule that controls several cellular processes, from the second messenger system to the induction of cell death. Type-2a Sarco/endoplasmic reticulum Ca^2+^-ATPase (SERCA2a) is a critical molecule for maintaining a balanced concentration of Ca^2+^ during the cardiac cycle, since it controls the transport of cytoplasmic Ca^2+^ to the sarcoplasmic reticulum (SR). The activity of this pump has been widely investigated, emphasizing its central role in the control of Ca^2+^ homeostasis and consequently in the pathogenesis of different cell types (Gianni et al., 2005; Park and Oh, 2013). Recent research has focused on the consequences of oxidative posttranslational modification (OPTM) of SERCA2a, such as Gαq-induced cardiac dysfunction (Lancel et al., 2010), ischemic injury-mediated irreversible SERCA2a modification, or age-related SERCA2a inactivity (Babusikova et al., 2012; Watanabe et al., 2016). Based on our previous research, we found that in addition to decreasing SERCA2a activity, cellular oxidative damage decreased the transcription of SERCA2a in CMECs. To determine whether SERCA2a undergoes OPTM, we used immunoprecipitation to observe the sulfonylation and tyrosine nitration of SERCA2a. Interestingly, the sulfonylation of cysteine 674 and the nitration of tyrosine at 294/295 in SERCA2a provided evidence of irreversible oxidation accompanied by cellular Ca^2+^ imbalance and TUNEL-positive cell death.

Another cytoplasmic Ca^2+^ storage organelle, the mitochondrion ([Ca^2+^]m), is filled with excess Ca^2+^ in some diseases, causing [Ca^2+^]m overload followed by severe side effects. Due to mitochondrial calcium overload, ATP depletion, oxidative stress, and disrupted mitochondrial matrix pH, a series of events leads to mPTP opening, which leads to mito-apoptosis via the release of cytochrome c to the cytoplasm and the activation of the intrinsic caspase pathway (Hausenloy and Yellon, 2013). Therefore, whether oxidatively modified SERCA2a-mediated [Ca^2+^]c imbalance triggers [Ca^2+^]m overload and mitochondrial damage needs further research. In our study, we found that CMEC hypoxic injury-induced [Ca^2+^]c and subsequent [Ca^2+^]m overload eventually led to mPTP opening and ΔΨm dissipation compared to the control. However, overexpression of SERCA2a or pretreatment with the [Ca^2+^]c chelator BAPTA restored mitochondrial function and morphology. Thus, we conclude that SERCA2a-dependent [Ca^2+^]c overload led to increased Ca^2+^ transport into mitochondria and subsequently caused excessive [Ca^2+^]m, which finally led to mitochondrial dysfunction and apoptosis. Schematic of the overall mechanism of heart ischemic injury in CMECs (Figure 7).

The article "Overexpression of SERCA2a Alleviates Cardiac Microvascular Ischemic Injury by Suppressing Mfn2-Mediated ER/Mitochondrial Calcium Tethering" was retracted in 2022. Reasons: compromised peer review; original data or images not available; concerns about the data.

**FIGURE 7:** Schematic of the overall mechanism of heart ischemic injury in CMECs.

Mitochondria/ER tethering is required for Ca^2+^ transfer from the SR to mitochondria. Strong evidence for the dependence of ER-mitochondrial Ca^2+^ microdomains on physical transorganelle linkage was provided by identifying the mitochondrial fusion protein (Mfn2) as a molecular tether that links SR to mitochondria (de Brito and Scorrano, 2008; Chen et al., 2012). There are two forms of Mfn: Mfn1 and Mfn2. Although studies have indicated that Mfn plays different roles in the heart and that its main function is far from clear, there is still some powerful evidence that shows that Mfn1 is more important as a mediator of mitochondrial fusion, while Mfn2 is important for mitochondria/ER tethering (Papanicolaou et al., 2012b). Moreover, published data revealed that cardiomyocyte-specific deletion of Mfn2 in normal mice increased mitochondrial size, which revealed its function in mitophagy (Papanicolaou et al., 2011, 2012a). A recent study highlighted the role of Mfn2 in the response of the adult heart to acute heart injury, but the results were unclear (Zhang and Yu, 2018). Other findings suggested that PGC-1α and Mfn2 constitute a regulatory pathway that plays a critical role in TNF-α-induced hepatic IRI (Li et al., 2014). MiR-497 inhibited cardiomyocyte apoptosis by downregulating the expression of Mfn2 in a mouse model of myocardial ischemic injury (Qin et al., 2018). Strong evidence proved that despite apparent mitochondrial dysfunction, hearts deficient in both Mfn1 and Mfn2 were protected against acute myocardial infarction due to impaired mitochondria/SR tethering (Hall et al., 2016). Adult Mfn2-deficient mice are protected against ischemic injury due to impaired mPTP opening (Tang et al., 2005). Therefore, based on previous studies, we decided to investigate the effect of cardiac Mfn2 knockout on microvessel endothelial cells in the context of heart ischemic injury. Our results indicated that disruption of the interaction between mitochondria and the SR plays an important role in reducing mitochondrial Ca^2+^ overload, subsequently attenuating mitochondrial oxidative stress and inhibiting mPTP opening [30].

The article "Overexpression of SERCA2a Alleviates Cardiac Microvascular Ischemic Injury by Suppressing Mfn2-Mediated ER/Mitochondrial Calcium Tethering" was retracted in 2022. Reasons: compromised peer review; original data or images not available; concerns about the data.

Furthermore, there have been no reports about the relationship between Mfn2 and SERCA2a inactivity in microvascular acute myocardial injury. We hypothesized that SERCA2a-induced [Ca^2+^]c imbalance is the upstream factor of Mfn2-mediated Ca^2+^ transport tethering. In our *in vivo* experiment, the results proved that either knockout of Mfn2 or overexpression of SERCA2a decreased heart infarction size, improved mitochondrial morphology, improved acute heart infarction indicators such as LDH, Troponin T, and CK-MB, restored myocardial contractile function, and maintained morphological structural integrity.

It is well-known that in addition to organelle tethering, Mfn2 is also involved in Parkin-mediated mitophagy to remove damaged mitochondria (Chan et al., 2011; Karbowski and Youle, 2011). We found that blocking Mfn2 expression not only reduced Ca^2+^ influx into mitochondria but also attenuated Parkin/PINK-dependent mitophagy and removal of damaged mitochondrial fragments. Although the Mfn2^KO^ group displayed prolonged and increased mitochondrial fragmentation, the expression of mito-apoptotic proteins and mitochondrial function were much better in the Mfn2^KO^ group than in the WT ischemic injury group.

In summary, we have shown that ablation of Mfn2 rendered the heart resistant to heart infarct injury and reduced cardiac microcirculatory damage. We proved that SERCA2a-dependent [Ca^2+^]c overload caused mitochondrial dysfunction and activated Mfn2-mediated [Ca^2+^]m overload. Knockout of Mfn2, the downstream target of SERCA2a, also suppressed fatal Drp-1-dependent mito-fission and Parkin/PINK-dependent mitophagy, which finally reduced heart ischemic injury in microvascular endothelial cells to some extent. In addition to impaired mitochondria/SR tethering, we provided a new mechanism for the role of Mfn2 inhibition during acute heart ischemia injury, which can be a novel strategy for microvessel cardioprotection.

## Data Availability Statement

The original contributions presented in the study are included in the article/supplementary material, further inquiries can be directed to the corresponding author/s.

The article "Overexpression of SERCA2a Alleviates Cardiac Microvascular Ischemic Injury by Suppressing Mfn2-Mediated ER/Mitochondrial Calcium Tethering" was retracted in 2022. Reasons: compromised peer review; original data or images not available; concerns about the data.

## Ethics Statement

The animal study was reviewed and approved by the Sixth Medical Center of Chinese PLA General Hospital.

## Author Contributions

YZ performed all the experiments. FT analyzed all the data. Both authors approved this submission.

## Conflict of Interest

The authors declare that the research was conducted in the absence of any commercial or financial relationships that could be construed as a potential conflict of interest.
